# Professional Quality of Life, Work-Related Stress, and Job Satisfaction among Nurses in Saudi Arabia: A Structural Equation Modelling Approach

**DOI:** 10.1155/2023/2063212

**Published:** 2023-01-31

**Authors:** Emad Shdaifat, Noha Al-Shdayfat, Najla Al-Ansari

**Affiliations:** ^1^Department of Community Health Nursing, College of Nursing, Imam Abdulrahman Bin Faisal University, P.O. Box 1982, City Dammam, Saudi Arabia; ^2^Community and Mental Health Nursing Department, Faculty of Nursing, Al Al-Bayt University, P.O. Box 130040, Mafraq, Jordan; ^3^Department of Nursing, King Fahd Hospital of the University, Al-Khobar, Saudi Arabia

## Abstract

**Objective:**

To examine the interrelated impacts of work-related stress, compassion satisfaction (CS), and job satisfaction on burnout (BO) and secondary traumatic stress (STS) among nurses using structural equation modelling (SEM).

**Methods:**

A cross-sectional design was used to survey 727 nurses at a teaching hospital in eastern Saudi Arabia. Three scales were used: the Quality of Life (ProQOL) scale, the Nursing Stress Scale (NSS), and the Job Satisfaction Survey (JSS). Data were analysed using SPSS and Analysis of Moment Structures (AMOS), and SEM analysis was conducted to confirm the interrelations among variables.

**Results:**

The final model had a good fit for the obtained data (*X*^2^ = 2.726, RMSEA = 0.032). Stress is directly related to BO and STS, and the following variables were directly related to STS: job satisfaction, BO, and CS. Lastly, BO mediated the relationship between stress and STS.

**Conclusion:**

It is crucial to analyze the effect of stress, CS, and job satisfaction which seems to have a positive and negative impact on nurses' BO and STS. Therefore, implementing a management strategy to manage stress and satisfaction can enhance nurses' quality of life, support the maintenance of positive attitudes, and enhance the standard of patient care.

## 1. Introduction

Nursing is fundamentally a caring science, and nurses are the frontline healthcare professionals who deliver the most personalized care for various service users [1]. Their work in hospitals is affected by numerous factors, including the amount of work delegated to them, the way they are managed by their supervisors, and their interactions or interrelationships at work as part of multidisciplinary healthcare teams and in liaising with service users [2]. Such work factors shape and influence their professional quality of life (QoL) either positively or negatively [3].

Due to the high rates of burnout (BO), absenteeism, and turnover among healthcare professionals worldwide, researchers have devoted increasing attention to exploring the status of professional QoL among caregivers and ways to improve it. Prolonged fatigue, emotional attrition, and a lack of perceived personal achievement can cause negative symptoms among employees [4]. On the other hand, the positive impact of altruism creates feelings of enjoyment from helping others, which is called compassion satisfaction (CS) [5]. According to Hegney et al. [6], self-efficacy beliefs, the feeling of being part of a community, and effective coping with different life situations are directly associated with CS. CS, obtained from caring and showing kindness and empathy for others, enhances the “professional and personal lives” of caregivers [7].

Compassion fatigue (CF) arises when nurses feel exhausted from delivering nonmedical aspects of nursing care to service users, which undermines their QoL as well as the quality of care they can provide [8]. CF encompasses two specific conditions, namely BO and STS [9]. It occurs gradually and is characterized by an inability to relate to and cooperate with people to whom they are entrusted to render service [10]. While BO originates from the person of the nurse experiencing stress, STS springs from caring for or attending to patients and families who experienced traumatic events first-hand. The trauma of patients and their families engenders anxiety, pressure, and other negative feelings among nurses during their interactions with service users [11].

Positive or negative impacts on professional QoL affect healthcare professionals' capacity to render safe, high-quality patient care [12]. In the midst of the plethora of nursing stressors, there are still factors in the job that render satisfaction to nurses, such as job environment, relations with colleagues and leaders, salary, promotion, security of employment, responsibility, and working hours [13]. Nevertheless, if a milieu of dissatisfaction outweighs these factors, nurses tend to leave their position, resulting in increased turnover, which represents a massive cost for healthcare systems worldwide [14].

Work-related stress, job satisfaction, and professional quality of life all play a substantial role in how well nurses accomplish their duties, which in turn affects patient outcomes and the effectiveness of the healthcare system [15]. Significant patient alienation, the development of negative attitudes toward job performance, a loss of compassion for patients, delays, and generally the substandard job performance are all effects of CF [16].

In order to understand the present aspect of nurses' experiences at work and to give a clear view of whether they are experiencing CF or CS, which affects the quality of patient care provided, it is important to explore nurses' professional QoL [17]. The nurse's level of stress could be measured to provide a baseline for developing intervention strategies to improve job satisfaction and orient nurses in relation to CS. The framework for enhancing the nursing workforce and services within the healthcare system could be strengthened by such knowledge. In order to alleviate work-related concerns for nurses and consequently enhance patient outcomes, nursing care quality, and health system effectiveness, considerable research in a variety of nursing contexts is necessary.

## 2. Literature Review

### 2.1. Study Variables

Healthcare is regarded as one of the most stressful occupations to work in [18], and nurses who work in a clinical setting are frequently confronted with extremely upsetting and stressful circumstances, such as deteriorating patient conditions and deaths [19, 20], which increase their burnout level and reduce their satisfaction with their work [21]. The National Institute for Occupational Safety and Health defines job stress as “the undesirable physical and emotional reactions that happen when the job specifications do not match the worker's capabilities, resources, or needs.” Workplace stress can result in poor wellbeing and even harm [22]. Burnout is characterized by exhaustion, cynicism, and inefficacy, described as three characteristics of a protracted response to ongoing workplace pressures [23]. Some studies have explored the relationships between work stress, job satisfaction, and CS with BO and STS [9, 24, 25]. Many studies have linked job stress to burnout [26–29] and job satisfaction [27, 30]. A prospective cohort study carried out by the Korea Nurses' Health Study (KNHS) among 10,305 nurses found a strong positive correlation between stress and burnout [31]. A meta-analysis found that stress had a weak positive correlation with burnout [32]. Among mental health nurses, it was found that burnout was positively correlated with job stress and was mediated by psychological capital [33].

In addition to relation between stress and BO, other researchers such as Back et al. confirmed the relation between nurses' stress and burnout with their job satisfaction and turnover intention [34, 35]. Locke defines job satisfaction as a pleasant or positive affection state that develops as a result of evaluating an individual's work experience [36]. According to the literature, job dissatisfaction is strongly linked to emotional exhaustion in healthcare workers, who are at high risk of burnout and work-related traumatic stress [37]. Among 620 nurses working in critical care units, job satisfaction was found to be associated with burnout [38]. Among critical care nurses in Saudi Arabia, Alharbi et al. [39] found that burnout is a predictor of job satisfaction. A study by Wu et al. involving 1464 banking professionals found that their job stress and burnout were mediated by job satisfaction [30]. In Greece, a study of 186 physicians and nurses reported that occupational stress was positively correlated with both burnout and STS [40].

Professional QoL (ProQOL) includes positive and negative traits. The influencing impacts or interacting dynamics between burnout, STS, and compassion fulfilment must be taken into account when talking about the work-related QoL of nurses [31]. CS is a positive emotion that shows the benefits of caring for others, which are also widely experienced by nurses. Working with patients and their families and obtaining good emotional benefits like satisfaction, joy, and hope results in CS [41]. However, in the course of caring for patients, nurses commonly experience STS, which is characterized by negative emotional responses (including fear and trauma) in response to witnessing negative events in the workplace. When nurses experience work-related trauma, usually a particular egregious occurrence, STS can occur [11].

The relation between ProQOL subscales was confirmed by Azizkhani et al. [42], who found that CS had a negative relationship with CF and BO. This result was proved by a meta-analysis which found that CS had a moderately negative correlation with burnout [32]. Zhang stated that reduced job satisfaction, compassion fatigue, and burnout are all directly correlated with the nursing profession's inherent stress and traumatic events [32]. Job satisfaction had a negative correlation with STS and CF [43, 44]. Several studies found that stress is related to or affects STS and CS [45, 46]. A study in Korea among 10,305 nurses found that both STS and CS both had a role in mediating the association between stress and burnout, which was found to be strongly mediated by stress [47].

Despite this tentative literature, there is still a dearth of studies confirming the association between ProQOL (CS, STS, and BO) subscales and work stress and job satisfaction, especially in particular contexts such as Saudi Arabia. The relation between stress and job satisfaction with ProQOL remains unclear; thus, this study explores mediators for this relationship.

We are not aware of any research that investigated the relation between CS, job satisfaction, and stress in the nursing field combined with BO and STS. As a result, this study is the first to connect CS, BO, stress, and job satisfaction into a unified model in order to better understand the dynamics of the working conditions as a whole and look at the BO as a mediator. In addition, this study is the first to identify such variables among Saudi Arabian nurses, and its findings serve as a standard for subsequent comparison.

This study provided an important opportunity to advance the understanding of the complex relationship between stress, CS, and job satisfaction in BO and STS, which was investigated in this study using SEM. We hypothesized that stress, CS, and JSS would have both direct and indirect impacts on BO and STS.

### 2.2. Study Context

Saudi Arabia is a high-income Eastern Mediterranean country [48], with USD 19,937 GDP per capita [49]. In 2021, the total population was 34.1 million, 36.4% of whom were non-Saudis [50]. The Ministry of Health (MOH), Other Government Healthcare (OGH), and Private Healthcare Sector (PHS) make up Saudi Arabia's healthcare system. The MOH provides the majority of healthcare services (60%), while the OGH and PHS each contribute 20%. Over 75% of all health spending in the Kingdom is state-funded, including the PHS [51].

In 2020, the total annual budget of the MOH was SAR 82 billion (USD 21.822 billion), which represents 8.2% of the general national budget. The ratios of hospital beds, physicians, and nurses per 10,000 people are 22.4, 27.2, and 54.9, respectively [52]. Since the MOH is the primary provider of medical services, a large portion of the population obtains care through the Ministry, which is in charge of delivering healthcare to the nation's residents [53]. Primary, secondary, and tertiary care are the three levels at which the MOH offers its public healthcare services. Primary healthcare services are the access point to additional healthcare facilities, whereas secondary and tertiary care are offered in general and specialty hospitals, accordingly.

## 3. Methods

### 3.1. Design and Setting

This cross-sectional, correlation study design was conducted at a university hospital in the Eastern Region of Saudi Arabia. The hospital has 491 beds and employs 727 nurses, providing services for 12,088 inpatients and 315,456 outpatients [54]. The study was part of a research project entitled “Assessing Compassion Satisfaction, Compassion Fatigue, Stress and Job Satisfaction Among Nurses.”

### 3.2. Sampling and Sampling Criteria

The sample comprised nurses from different units at all shifts in both critical and noncritical units. Participants from critical units represented MICU, SICU, Burn Unit, CCU NICU, and PICU. The purposive sampling method was used; inclusion criteria stipulated that participants had to be registered nurses (RNs) with at least a diploma, employed as staff nurses in hospitals. Nurses with less than six months' experience were excluded from the study.

The survey was administered through the survey program QuestionPro (http://www.questionpro.com), a service for conducting online research. Survey links were sent via email to 727 full‐time RNs who had a diploma, an associate, a baccalaureate, or a master's degree and had been working in their current unit for more than six months.

### 3.3. Survey Instruments

The survey was in the English language (the professional language of healthcare professionals in Saudi Arabia) and consisted of four parts. The first part gathered nurses' demographic and professional variables. The second part evaluated CS and CF using the Professional Quality of Life (ProQOL) scale. The third part evaluated stress level using the Nursing Stress Scale (NSS), and the final part evaluated job satisfaction using the Job Satisfaction Survey (JSS).

ProQOL evaluates CS and CF with 30 Likert-type items, with responses ranging from 1 (never) to 5 (very often). ProQOL is divided into three scales, CS, BO, and STS. Participants are asked to evaluate their experience with patients over the last 30 days [55]. The average score of CS, BO, and STS is 50, and alpha scale reliability was 0.88, 0.75, and 0.81, respectively [11]. In this study, the STS, CS, and BO dimensions have alpha scale reliability values of 0.86, 0.84, and 0.77, respectively. The Kaiser–Meyer–Olkin (KMO) value was 0.87, above the recommended value of 0.6 [56, 57], and Bartlett's test of sphericity [58] achieved statistical significance. Convergent validity was assessed using the average variance extracted (AVE), with a value of 0.5.

The NSS is widely used to measure nurses' stress. It includes 34 Likert-type items ranging from 0 (never) to 4 (very frequent), with a Cronbach's alpha coefficient of 0.89. The scale is divided into seven subscales: death and dying, conflict with physicians, inadequate preparation, lack of support, conflict with other nurses, workload, and uncertainty concerning treatment [59]. In our study, alpha scale reliability was 0.94. The KMO value was 0.89, above the recommended value of 0.6 [56, 57], and Bartlett's test of sphericity [58] reached statistical significance. Convergent validity was assessed using the AVE, with a value of 0.4.

The JSS is used to evaluate employees' attitudes about their job. It includes 36 items to evaluate nine dimensions of job satisfaction: pay, promotion, supervision, fringe benefits, contingent rewards, operating conditions, coworkers, nature of work, and communication. The scale uses Likert-type answers, ranging from 1 (disagree very much) to 6 (agree very much) [60]. In this study, the alpha scale reliability was 0.88. The KMO value was 0.83, above the recommended value of 0.6 [56, 57], and Bartlett's test of sphericity [58] attained statistical significance. Convergent validity was assessed using the AVE, with a value of 0.5.

### 3.4. Ethical Consideration

Approval to carry out the study was obtained from the Institutional Review Board at the university where the research team is established. The invitation email sent to participants explained the voluntary nature of participation and that they could refuse to participate or subsequently withdraw prior to submitting the completed questionnaire. They were informed that their answers would remain anonymous and would only be used for academic purposes and that no personal identifying information was included in the survey. By completing the online survey and submitting it, they indicated that they understood their rights and voluntarily consented to participate.

### 3.5. Data Collection

The questionnaire was sent to nurses working on all shifts (morning, evening, and night) via their official email accounts. Data collection took place over three months.

### 3.6. Data Analysis

Questionnaire data were transferred from QuestionPro as an SPSS file. Data were stored and analysed using SPSS version 22.0 and Analysis of Moment Structures (AMOS) version 21. The questionnaires used in the study were assessed for reliability and validity in terms of internal consistency (Cronbach's alpha), and convergent validity was assessed using AVE, as explained above. Categorical variables were presented by frequencies and percentages, while continuous variables were presented by mean and standard deviation (SD). Pearson correlation analysis was used to evaluate the relation between ProQOL, stress, and job satisfaction. An alpha level of *p* < 0.05 was set as significant in all analyses. SEM was used to test the relations between the study variables.

SEM is a type of multivariate analysis which was applied to check the theoretically built model that includes the domains of CS, BO, stress, and job satisfaction, with STS domains. The chi-square statistic provides a test of the null hypothesis that the theoretical model fits the data. The criteria for model fit were a relative chi-square statistic less than or equal to 2.0, a goodness-of-fit index (GFI) statistic equal to or greater than 0.95, an adjusted goodness-of-fit index (AGFI) statistic equal to or greater than 0.90, a comparative fit index (CFI) equal to or greater than 0.90, and a root mean square error of approximation (RMSEA) less than or equal to 0.8. A higher Parsimony ratio (PRatio) suggests that the model is more parsimonious. Total, direct, and indirect effects of stress, job satisfaction, CS, and BO on STS were calculated using the standardized regression weights of each pathway.

## 4. Results

### 4.1. Participant Characteristics

The response rate was 47.7%.  Table 1 shows that the majority of the participants were female (89.3%), married or divorced (61.7%), had BSN or MSN qualifications (81.6%), were non-Saudis (91.6%), and were working in rotational shifts (74.6%). The mean age of participants was 34.8 (SD7.9) years old, and their experience was 9.8 (SD6.7) years.

### 4.2. Correlation Coefficients

A Pearson product-moment correlation was performed to examine the relationships between STS, CS, BO, stress, and job satisfaction. STS has a moderately positive relation to BO (*r* = −0.53, *p* < 0.01), which is stronger than its relationship with stress (*r* = 0.44, *p* < 0.01), and the lowest relation is with job satisfaction (*r* = 0.13, *p* < 0.05). STS was moderately negatively related to CS (*r* = −0.23, *p* < 0.01).

CS has a weak negative relation with BO (*r* = −0.11, *p* < 0.05) and stress (*r* = −0.26, *p* < 0.01) and a positive correlation with job satisfaction (*r* = 0.23, *p* < 0.01). BO had a moderately positive relation with stress (*r* = 0.48, *p* < 0.01) and a weak one with job satisfaction (*r* = 0.09, *p* < 0.05). Finally, stress had a weak positive relation with satisfaction (*r* = −0.02, *p* < 0.05) (Table 2).

### 4.3. Final Model

The final model and goodness-of-fit indices are presented in Figure 1. The measures of model fitness were as follows: chi-square for the goodness-of-fitness test (*x*^2^ = 2.726, d*f* = 2, *p* = 0.256), relative chi-square (1.363), GFI (0.997), AGFI (0.977), CFI (0.997), PRatio (0.200), and RMSEA (0.032). All indices indicate that the present model fits the data.

### 4.4. Significant Relationships between Observed Variables

The results of the significant relationships between stress, job satisfaction, BO, CS, and STS are shown in Table 3. Stress is directly related to BO (*b* = 0.17; *p* < 0.001) and STS (*b* = 0.17; *p* < 0.001). Job satisfaction is directly related to STS (*b* = 0.13; *p* < 0.004). BO and CS are directly related to STS (*b* = 0.40; *p* < 0.001, and *b* = −0.16; *p* < 0.001, respectively).

### 4.5. Mediating Factors

Table 4 shows the direct and indirect effects of the independent variables on the dependent variables. BO was a mediator between stress and STS. Stress was directly related to BO (*B* = 0.48). On the other hand, stress was directly and indirectly related to STS (mediated by BO, total *B* = 0.40). Job satisfaction was directly related to STS (*B* = 0.13), and CS was directly related to STS (*B* = −0.16).

## 5. Discussion

The current study findings provide crucial insights into exploring interrelationships among various components of the ProQOL, thereby increasing understanding of these components. This provides stakeholders with a comprehensive picture of nurses' ProQOL, in order to consider proper management strategies to improve their working conditions, which in turn would contribute to enhancing their ProQOL, improving the quality of care they provide, and increasing healthcare system efficiency.

The results of this study indicate that CS is inversely associated with STS. Unexpectedly, the results indicated that CS and BO were not significantly associated. In addition, stress was associated directly and indirectly through BO with STS. Consequently, BO was a mediator in the relationship between stress and STS. Another important finding is that job satisfaction was directly associated with STS.

The most important finding in ProQOL was that CS was directly and inversely associated with STS; thus, increased CS predicts lower STS. Preserving nurses' compassion for their job significantly influences their practice (i.e., the quality of service delivery). Many studies explored the relationship between CS and the levels of STS they may experience. This finding was incongruent with many studies [7, 61, 62]; only one study was found which reported that CS is positively correlated with STS [63]. This may be attributable to hospital settings having a significant impact on the CS level among nurses, whereby nurses who receive positive support in their job do not complain about any significant fears. Nurses are more likely to enjoy dealing with patients who need them and are appreciative of their help [11].

Contrary to expectations, CS and BO were not significantly associated. The reason behind this might be that the participants have coping mechanisms to deal with stressful working conditions. Also, most of the nurses who participated in our study were non-Saudis, which means that they are essentially economic migrants primarily motivated to work abroad in a challenging environment due to financial motivations. Consequently, they may accept hard and stressful working conditions in order to preserve their financial resources, especially during the COVID-19 pandemic, in which many workers have lost their jobs all over the world. Put simply, they are primarily motivated by the economic goal of supporting their socioeconomically deprived families in their homelands and not by a quest for their own personal, professional, or individual satisfaction.

Our results are in line with a previous study, which found that CS was not associated with CF (BO and STS) [64]. However, this is inconsistent with other literature, as many studies revealed a significant association between CS and BO. For example, a study conducted in India to explore healthcare providers' ProQOL and associated factors found a negative correlation between CS and BO and a positive correlation between BO and STS [65]. A recent study conducted in Jordan to find out the level of CF, BO, and CS among oncology nurses showed that BO was significantly related to CF [66]. Similarly, a negative association was found between CS and BO [67].

In addition, stress was associated directly and indirectly through BO with STS, so increased stress predicts increased BO and STS. Previous studies confirmed that higher stress is linked with high CF and low CS [8]. Job stress is mainly connected with physical and psychological stress among nurses [68]. Moreover, stress is linked with higher BO and lower levels of CS [69]. According to Fiore, extended stress can lead to BO, health issues, and turnover. Thus, stress can negatively impact [70] professional QoL and increase attrition among the nursing workforce. Numerous studies have demonstrated that stress has direct and indirect relationships with BO, STS [31, 71], and CF [19]. Surprisingly, Itzhaki et al. [68] found that work stress was not associated with STS. This may be due to the high number of female nurses among participants; usually, females have poorer health and lower QoL than males [72]. In addition, during the peak of the COVID-19 pandemic, healthcare providers had higher levels of CF and stress and lower CS [8].

We found that BO mediates the relationship between stress and STS, corresponding with a study which found that STS and CS mediate the relationship between stress and BO [31]. Other study results reported that STS is predicted by high scores of BO and CF [73]. Nevertheless, the interrelations between BO, STS, and stress are expected. CF has been found to mediate the relation between stress and CS [19]. Stress was associated with BO and mediated by STS [31]. Nurses lacked time to care for patients because their workload experienced high STS [45].

Moreover, job satisfaction was directly associated with STS, whereby increased job satisfaction increases STS. Our finding was in keeping with previous literature [62, 72, 74, 75]. In addition, Ogińska-Bulik et al. [76] found that the main predictor of STS symptoms is job satisfaction. Job satisfaction can be difficult to assay among nurses, as nurses can be highly effective at biomedical aspects of nursing care delivery, taking their roles seriously, while experiencing reluctance or even fear of engaging with service users and with other healthcare staff. Nurses in this category benefit from encouragement to build on their feelings of altruism and beliefs that they are providing good quality care to their patients [11]. It is recommended to establish an efficient management plan to lessen nurses' BO in a way that reduces stress and increases CS.

## 6. Conclusion

This study examined the effect of stress, CS, and job satisfaction on BO and STS. One of the more significant findings to emerge from this study is that CS is inversely associated with STS; thus, increased CS predicts lower STS. Unexpectedly, CS and BO were not significantly associated. In addition, stress was associated directly and indirectly through BO with STS; thus, stress predicts increased BO and STS. Therefore, BO mediates the relationship between stress and STS. Moreover, job satisfaction was directly associated with STS.

The findings of this study have a number of implications, the most obvious of which is that nursing managers should be more aware of the factors affecting CS, BO, and STS, and they should seek to evaluate the level of stress and satisfaction. Nurses provide medical, psychological, and spiritual care for their patients, yet they themselves can be affected negatively by their responsibilities and interactions with patients. Consequently, nurses who receive the necessary help and support will be in a better position to provide care for patients. Managers must be concerned about the negative impacts on care due to nurses suffering from BO and STS and seek to reduce these effects by fostering more supportive working conditions and environments, which improve employee satisfaction, increase quality of care, improve patient outcomes, and reduce health system costs and inefficiencies. Positive impacts of caring, such as CS, should be deliberately promoted in inspirational and motivational ways. Hospital managers should design interventions to reduce BO, STS, and stress and to improve CS and job satisfaction through education on using coping strategies, and they should offer more healthy working conditions. Nurse managers and policymakers should emphasize forming healthy and stress-free working conditions to provide a better quality of services.

## 7. Limitations

Several limitations of this study need to be acknowledged. First, the study was conducted at a single institution, and participants were restricted to nurses in one teaching hospital, which limits the generalizability of results. Future studies are encouraged to involve nurses from other health sectors. In addition, the data collection used a self-administered questionnaire to reflect nurses' feelings, which can vary over time. Also, future studies should focus on working conditions and other factors that can affect ProQOL.

Our study focused on stress, job satisfaction, and burnout, which are intrinsically related to nursing work, but future research should explore differentiating between sources of stress (e.g., work-related or family-related). Personal stressors such as family problems, financial status, and difficult relationships should be investigated in relation to work-related stress, burnout, job satisfaction, and nurses' overall health [77]. More research is required to address the underlying causes of nurse dissatisfaction [78].

Cross-sectional surveys, whereby each participant's exposure and outcome are determined at the same time, make causal inferences difficult. Random and large-scale sampling is needed to ensure that each person has a similar chance of being included in the study and that the recruited sample represents the study population. This limitation necessitates additional longitudinal research into the mediating effects between ProQOL, stress, and job satisfaction among nurses [79].

Although the findings should be interpreted with caution, this study has several strengths, including the combination of stress and job satisfaction in the ProQOL framework as one construct because of the interaction between those factors. Moreover, involving nurses from different units helps represent both the critical and noncritical care units, which are represented in the results. It is recommended that further research implement this approach in different clinical sites, and a longitudinal study evaluating ProQOL over time would be very useful.

## Figures and Tables

**Figure 1:** Significant pathways of the final model and goodness-of-fit indices. d*f* = degree of freedom; GFI = goodness-of-fit index; AGFI = adjusted goodness-of-fit index; CFI = comparative fit index; Pratio = Parsimony ratio; RMSEA = root-mean square error of approximation.

**Table 1:** Demographic characteristics of nurses (*n* = 347).

Variable	Frequency	Percent	

Gender			
Female	310	89.3	
Male	37	10.7	
Marital status			
Single	133	38.3	
Married/divorced	214	61.7	
Education level			
Diploma	64	18.4	
BSN or MSN	283	81.6	
Nationality			
Saudi	29	8.4	
Non-Saudi	318	91.6	
Unit			
Critical units	162	46.7	
Non critical units	185	53.3	
Shift work			
Fix (A, B, C)	88	25.4	
Rotational	259	74.6	

	Mean (SD)	Max.	Min.
Age	34.8 (7.9)	24	60
Experience	9.8 (6.7)	1	34

**Table 2:** Pearson correlation coefficient matrix of the measured variables.

	STS	CS	Burnout	Stress	Satisfaction
STS	1				
CS	−0.23^*∗∗*^	1			
Burnout	0.53^*∗∗*^	−0.11^*∗*^	1		
Stress	0.44^*∗∗*^	−0.26^*∗∗*^	0.48^*∗∗*^	1	
Satisfaction	0.13^*∗*^	0.23^*∗∗*^	0.09	0.02	1

^*∗∗*^Correlation is significant at the 0.01 level. ^*∗*^Correlation is significant at the 0.05 level.

**Table 3:** Relationship between independent and dependent variables.

Independent variable		Dependent variable	*B*	*b*	*t* stat.	*p* value
Stress	⇢	Burnout	0.48	0.17	10.07	<0.001
Stress	⇢	STS	0.21	0.17	4.06	<0.001
Job satisfaction	⇢	STS	0.13	0.10	2.89	<0.004
Burnout	⇢	STS	0.40	0.91	8.10	<0.001
CS	⇢	STS	−0.16	−0.22	−3.49	<0.001

*B* = standardized regression coefficient; *b* = unstandardized regression coefficient (95% CI of unstandardized regression coefficient).

**Table 4:** Total, direct, and indirect effects of independent variables on dependent variables.

Dependent variable	Effect^a^	Independent variable		
		Stress	Job satisfaction	CS
Burnout	Total	0.48	0.00	0.00
	Direct	0.48	0.00	0.00
	Indirect	0.00	0.00	0.00

STS	Total	0.40	0.13	−0.16
	Direct	0.21	0.13	−0.16
	Indirect	0.19	0.00	0.00

^a^Standardized regression weight (*B*).

## Data Availability

Data are available from the corresponding authors upon reasonable request.
